The article "MIG-7 and phosphorylated prohibitin coordinately regulate lung cancer invasion/metastasis" was retracted in 2019. Reasons: fabricated or falsified data; fabricated or falsified images; an official misconduct investigation; misconduct by an author.

# MIG-7 and phosphorylated prohibitin coordinately regulate lung cancer invasion/metastasis

**DOI:** 10.18632/oncotarget.2804

**Published:** 2014-11-16

**Authors:** Ming-Yi Ho, Chi-Ming Liang, Shu-Mei Liang

**Affiliations:** ^1^ Genomics Research Center, Academia Sinica, Taipei, Taiwan, ROC; ^2^ Agricultural Biotechnology Research Center, Academia Sinica, Taipei, Taiwan, ROC

**Keywords:** growth factors, migration inducting gene-7 (MIG-7), prohibitin (PHB), COX-2/PGE2, lung cancer invasion/metastasis

## Abstract

Growth factors and COX-2/PGE2 enhance lung cancer invasion/metastasis via PI3K/Akt and RAS/Raf. Here, we explored their mechanism of action further. We found first that higher levels of migration inducting gene-7 protein (MIG-7) and PHB phosphorylated at threonine 258 (phospho-PHB^T258^) are positively correlated with advanced stages of human lung cancer in tissue microarray. PGE2 or growth factors such as EGF, HGF and IGF-1 increased complex formation of phospho-PHB^T258^ with Ras, phospho-Akt^S473^, phospho-Raf-1^S338^, MEKK1 and IKKα/β^S176/180^ in the raft domain transiently within 1 hour and MIG-7 in the cytosol 12-24 hours later. Association of phospho-PHB^T258^ with MEKK1 but not MEKK3 activates IKK/IκB/NF-κB and MEK/ERK to increase cellular COX-2/PGE2 and an E-cadherin suppressor Snail leading to enhancement of epithelial-mesenchymal transition (EMT) and lung cancer migration/invasion. MIG-7, on the other hand, was induced by growth factors and PGE2 via Akt/GSK-3β in a phospho-PHB^T258^ independent manner. MIG-7 increased two E-cadherin suppressors ZEB-1 and Twist to enhance EMT and cancer migration/invasion. Downregulating phospho-PHB^T258^ and MIG-7 had an additive effect on attenuating lung cancer invasion/metastasis and prolonging the survival of xenograft mice. Phospho-PHB^T258^ and MIG-7 may thus play complementary roles in the initiation and sustainment of the effects of growth factors and COX-2/PGE2 on cancer invasion/metastasis.

## INTRODUCTION

Metastasis is the major cause of lung cancer treatment failure and mortality [1-3]. Although there are currently more than 1000 clinical and preclinical trials and about 350 of them deal with advanced lung cancer, no therapeutic approach targeting one single pathway provides impressive results in terms of prolonging patient survival [4]. Exploration of a better drug target and rational design of combinational treatment of multiple pathways are thus urgently needed.

Migration inducting gene-7 (MIG-7) protein, a potential mediator of metastasis [5-7] is functionally associated with COX-2/prostaglandin E2 (PGE2)-induced lung cancer metastasis through phosphorylation of Akt and glycogen synthase kinase-3 β (GSK-3β), activation of wnt/β-catenin/TCF-4/LEF-1 signaling and decrease in the activity of protein phosphatase 2A (PP2A) [8]. Knockdown of MIG-7, however, causes only partial (30-60%) rather than complete attenuation of lung cancer epithelial-mesenchymal transition (EMT) and migration/invasion/metastasis [8].

Another potential mediator of lung cancer metastasis is prohibitin phosphorylated at threonine 258 (phospho-PHB^T258^) [9]. Stable expression of phospho-PHB^T258^ in the plasma membrane of CL1-0 human lung cancer cells enhances EMT and invasion/metastasis. In addition, phospho-PHB^T258^ has been shown to associate with Raf-1 to enhance Raf-1 activation and the invasive capability of cancer cells [9]. The functional interrelationship between phospho-PHB^T258^ and MIG-7 in lung cancer invasion/metastasis remains, nonetheless, largely unexamined.

Poor lung cancer prognosis is frequently associated with overexpression of COX-2/PGE2 [10-13]. A variety of scenarios, notably smoking, nicotine and long-term inflammation, result in high levels of COX-2/PGE2 that induce tumor angiogenesis and augment cancer invasiveness [14-18]. Although MIG-7 has been shown to regulate COX-2/PGE2-mediated lung cancer metastasis, the influence of phospho-PHB^T258^ on the actions of COX-2/PGE2 is unclear.

Growth factors such as EGF, HGF and IGF-1 increase the matrix metalloproteinase (MMP) activity to enhance migration/invasion of lung cancer cells [19]. Aberrant activation of EGF and IGF-1 receptor signaling enhances EMT and lung cancer invasion/metastasis [20, 21]. Whether COX-2/PGE2, phospho-PHB^T258^ and MIG-7 are cellular mediators for the effects of growth factors on lung cancer invasion has not been fully elucidated.

In this study, we found that the levels of plasma membrane-associated PHB and MIG-7 were positively correlated with advanced stages of cancers in human lung tumor tissues. PGE2 and growth factors notably EGF, HGF or IGF-1 increased phosphatidylinositol-(3,4,5)-triphosphate (PIP3) and phospho-PHB^T258^ in membrane rafts leading to transient association of Ras with phospho-Akt^S473^ within 1 hour. This transient association enhanced colocalization of MEKK1 and phospho-IKKα/β^S176/180^ in membrane rafts resulting in elevation of IKKα/β/IkB/NF-kB activation and cellular COX-2/PGE2 expression. PGE2, EGF, HGF or IGF-1 also increased cytosolic MIG-7 level that occurred 12-24 hours later and sustained for a long period of time. We also found that phospho-PHB^T258^ and MIG-7 acted coordinately to increase distinct E-cadherin suppressors and promote EMT and lung cancer invasion/metastasis. The critical role of phospho-PHB^T258^ and MIG-7 in cancer invasion/metastasis was further substantiated by downregulation of MIG-7 and/or phospho-PHB in a human lung cancer xenograft mouse model.

## RESULTS

### Levels of MIG-7 protein and plasma membrane-associated PHB correlate with advanced stages of cancers in human lung tumor tissues

We have recently analyzed the level of MIG-7 in a human lung carcinoma tissue microarray and found a positive correlation between MIG-7 and advanced stages of lung cancer [8]. Here, we further analyzed the level of plasma membrane-associated PHB in tumor and normal lung tissues and examined its correlation with MIG-7 and advanced stages of lung cancer. Our results showed that like MIG-7, the median levels of membrane-associated PHB were higher in lung cancer (T) than normal (N) lung tissues (*P* < 0.001); in tumor that invaded into subserosa or other organs (T3 + T4) versus tumor that invaded submucosa or muscularis propria (T1 + T2) (*P* < 0.01); in cancers with lymph node involvement (N1 + N2) versus cancers without lymph node involvement (N0) (*P* < 0.001); and in stage II/III/IV versus stage I lung cancer (*P* < 0.001) (Figure 1A). Moreover, the tumors with more MIG-7 proteins also tended to exhibit higher plasma membrane-associated PHB scores (Spearman correlation coefficient r = 0.4628; *P* < 0.0001; Figure 1B).

**Figure 1:** The levels of MIG-7 protein and plasma membrane-associated PHB positively correlates with advanced stages of cancers in human lung tumor tissues Lung tissue sections from a human lung carcinoma microarray were immunostained with anti-PHB and anti-MIG-7 antibodies, respectively. (A) The percentage of positive cells and intensity of plasma membrane-associated PHB in each tissue sample were scored as described in Materials and Methods. More membrane-associated PHB was found in cancers (T; n =89) than normal tissues (N; n = 10); in T3+T4 cancers (n = 28) versus T1+T2 cancers (n = 61); in cancers with lymph node involvement (N1+N2; n = 44) versus those without lymph node involvement (N0; n = 45); and in stage II+III+IV ( n = 51) versus stage I lung cancer (n = 38). Data are expressed as medians relative to each group of tissues. **P < 0.01, ***P < 0.001. (B) Scatter plot was generated by plotting the levels of MIG-7 versus those of membrane-associated PHB (left panel; Spearman correlation = 0.4628, *P* < 0.0001). The representative lung tumor sections were examined at ×200 magnification for MIG-7 and membrane-associated PHB (right panel).

### Growth factors and PGE2 increase PIP3 and phospho-PHB^T258^ in membrane raft as well as MIG-7 in cytosol in distinct temporal patterns

High levels of COX-2/PGE2 and growth factors notably EGF, HGF and IGF-1 enhance EMT and cancer invasion/metastasis [10-13, 19-21]. To examine whether these effects are via MIG-7 and phospho-PHB^T258^ - the active PHB molecule in membrane rafts [9], we treated lung cancer cells with EGF, HGF, IGF-1 and PGE2, respectively. Our results showed that PIP3, an inositol phospholipid known to activate Akt/PHB signaling pathway [9, 22, 23], was increased by EGF, HGF, IGF-1 and PGE2 in a concentration dependent manner (Figure 2, left panels). The level of PIP3 reached a plateau at 60 min and then declined (Supplementary Figure 1). This transient increase in PIP3 was accompanied with an increase of phospho-Akt^S473^ and phospho-PHB^T258^ (Figure 2 middle panels). EGF, HGF, IGF-1 and PGE2 also increased the levels of MIG-7, COX-2 and PGE2, but the increase of MIG-7, COX-2 and PGE2 was found not within 60 min but at 12-24 hours [8]; Figure 2 middle and right panels).

**Figure 2:** EGF, HGF, IGF-1 and PGE2 increases PIP3, phospho-Akt phospho-PHB, MIG-7, COX-2 and cellular PGE2 Lung cancer cells (A549, CL1-0 and CL1-5; 2 × 10^5^/mL) were treated with or without EGF, HGF, IGF-1 and PGE2 for 24 hours at concentrations as indicated. Cells were then harvested and PIP3 levels in phospholipid fraction were determined by ELISA (left panels). Data represent means ± SD of 3 independent experiments; *, *P* < 0.05 by t test. Proteins of lung cancer cells were determined by immunoblotting. The levels of COX-2 and MIG-7 were determined 24 hours after treatment while all others were determined 1 hour after treatment (middle panels). Blots are representative of 3 independent experiments. The cellular contents of PGE2 were determined by ELISA (right panels). Data represent means ± SD of 3 independent experiments; ns, not significant; *, *P* < 0.05 by t test.

### PIP3-mediated increase of COX-2/PGE2 is positively correlated with increase of phospho-PHB^T258^ and MEKK1

Although PIP3 activates integrin-linked kinase (ILK) and Akt, notably Akt/IKKα/β/IκB/NF-kB pathway, to induce COX-2 [22-24], the involvement of PHB in this effect of PIP3 is unclear. We found that PIP3-mediated increase of phospho-NF-kB p65^S536^, COX-2 and PGE2 was positively correlated with an increase in not only phospho-Akt^S473^, phospho-Akt^T308^, and phospho-IKKα/β^S176/180^ but also phospho-PHB^T258^ in membrane rafts (Supplementary Figure 2A and 2B).

To further explore the functional involvement of active Akt and PHB with PIP3-mediated enhancement of IKKα/β/IκB/NF-kB signaling, we transfected lung cancer cells with dominant negative Akt (*Akt-DN*), dominant active Akt (*Akt-DA*) and then treated the cells with PIP3. Our results showed that PIP3 increased phospho-PHB^T258^, phospho-IKKα/β^S176/180^, phospho-NF-kB p65^S563^ and COX-2 in an Akt-dependent manner (Figure 3A). Since Ras regulates cellular functions via PI3K/Akt and PHB [9], we examined which PIP3-induced proteins in membrane raft were immunoprecipitated by anti-Ras antibodies. We found that PIP3 increased the association of Ras with not only phospho-PHB^T258^ and phospho-IKKα/β^S176/180^ but also mitogen-activated protein kinase/ERK kinase kinase-1 (MEKK1) in an Akt dependent manner (Figure 3B).

**Figure 3:** PIP3 increases phospho-PHB^T258^, phospho-IKKα/β^S176/180^, phospho-NF-kB p65^S536^ and COX-2 as well as formation of Ras/Raf/PHB/MEKK1/IKK complex in a phospho-Akt dependent manner (A) dominant negative Akt (*Akt-DN*) attenuated the effects of PIP3 on not only COX-2 but also phosphorylation of Akt, PHB, IKKα/β and NF-kB. Lung cancer cells (A549 and CL1-0; 2 × 10^5^/mL) transfected with empty vector (EV), dominant active-(DA) or dominant negative-(DN) Akt for 48 hours were treated with or without PIP3 (5 μM) for 24 hours as indicated. The protein levels were determined by immunoblotting. (B) lung cancer cells (2 × 10^5^/mL) transfected with or without *Akt-DN* plasmid for 48 hours were treated with 5 μM PIP3 for 24 hours as indicated. The membrane raft fractions were immunoprecipitated with anti-Ras antibodies, and the immunoprecipitated proteins were detected by immunoblotting. Caveolin-1 and clathrin heavy chain (HC) protein served as membrane raft and non-raft markers, respectively. (C and D), cells were transfected with plasmids *pBio-PHB*, *pD-PHB* or empty vector (*pBio-vector* and *pD-vector*) for 48 hours, as indicated. The cell extracts were immunoprecipitated with anti-IKKα/β or anti-PHB antibodies and the immunoprecipitated proteins were detected by immunoblotting. Blots are representative of 3 independent experiments.

IKK/IκB/NF-kB signaling has been shown to be regulated differentially by MEKK1 and NF-kB inducing kinase (NIK) [25]. Whether PIP3-mediated activation of IKK/IκB/NF-kB signaling requires MEKK1 and/or NIK is largely unclear. To gain insight into the potential involvement of active PHB, MEKK1 and/or NIK in the Ras/Raf and IKKα/β/IκB/NF-kB signaling, lung cancer cells were transfected with *pBio-PHB* or *pD-PHB* to generate biotin-labeled or plasma membrane-bound active PHB, respectively, and then co-immunoprecipitated with anti-IKKα/β or anti-PHB antibodies (Figure 3C and 3D). Our results revealed that phospho-PHB^T258^ in the raft domain was associated with Ras, phospho-Akt^S473^, phospho-Raf-1^S338^, IKKα/β^S176/180^ and MEKK1 but not with NIK or MEKK3 (Figure 3C and 3D). Moreover, generation of active PHB by *pBio-PHB* or *pD-PHB* increased MEKK1 and phosphorylated IKKα/β in the raft domain as well as phospho-NF-kB p65^S536^ and COX-2 in the non-raft fraction (Supplementary Figure 3A). These results demonstrated that PIP3-mediated enhancement of IKKα/β/IκB/NF-kB signaling and COX-2 requires active PHB and MEKK1 but not NIK.

To examine whether MEKK1 is upstream or downstream of PHB, IKKα/β^S176/180^ and NF-kB p65^S536^, cells were transfected with wild-type (wt) and dominant negative MEKK1 plasmid (*pMEKK1-DN*) and then treated with or without PIP3. Transfection with *MEKK1-wt* or *MEKK1-DN* did not affect the levels of phospho-Akt or phospho-PHB, indicating that Akt/PHB is upstream of MEKK1. PIP3-mediated phosphorylation of IKKα/β^S176/180^ and NF-kB p65^S536^ as well as expression of COX-2, on the other hand, are downstream targets of MEKK1 as they were attenuated by downregulating MEKK-1 with *pMEKK1-DN* (Supplementary Figure 3B).

### Phospho-PHB^T258^ in membrane raft is indispensable for PIP3-mediated increase of phospho-IKKα/β^S176/180^, phospho-NF-kB p65^S536^ and COX-2

To confirm the critical role of phospho-PHB^T258^ in the PIP3-mediated increase of MEKK1, phospho-IKKα/β^S176/180^, phospho-NF-kB p65^S536^ and COX-2, we knocked down PHB with PHB siRNA (*siPHB*) and tested whether phospho-PHB mutants with site-directed mutation at T258 and Y259 could reverse the inhibitory effects of *siPHB* as the wild type phospho-PHB. Downregulation of PHB with *siPHB* attenuated PIP3-mediated increase in phospho-IKKα/β^S176/180^, phospho-NF-kB p65^S536^ and COX-2 (Supplementary Figure 4A). The inhibitory effect of *siPHB* was not reversed by *pBio-PHB^T258I/Y259F^* double mutant (T/Y), but was reversed by *pBio-PHB* (wt) that generated biotin-labeled active phospho-PHB^T258^ (Supplementary Figure 4A). Analysis of protein levels in the raft and non-raft domains further demonstrated that neither *pD-PHB ^T258I^* nor *pD-PHB^Y259F^* mutant plasmid increased the level of MEKK1 or phospho-IKKα/β^S176/180^ in the raft domain (Supplementary Figure 4B). Co-immunoprecipitation with anti-hemagglutinin (HA) antibodies that recognize N-terminal epitope of HA tagged to D-PHB [9] showed that *pD-PHB (wt)* but not *pD-PHB^T258I^* or *pD-PHB^Y259F^* was associated with phospho-IKKα/β^S176/180^ (Supplementary Figure 4C). Moreover, only *pD-PHB (wt)* but not *pD-PHB^T258I^* or *pD-PHB^Y259F^* increased phospho-NF-kB p65^S536^ and COX-2 in the lysate (Supplementary Figure 4C).

### Phospho-PHB^T258^ and MIG-7 play distinct roles in enhancement of EMT

Cancer cell migration/invasion and metastatic capability are strongly associated with EMT [8, 9]. Although both phospho-PHB^T258^ and MIG-7 increase E-cadherin suppressors such as Snail, ZEB-1 or Twist to enhance EMT [8, 9], downregulation of either phospho-PHB^T258^ or MIG-7 causes only partial (30-60%) rather than complete attenuation in lung cancer EMT [8, 9]. To further understand this phenomenon and delineate the functional relationship between phospho-PHB^T258^ and MIG-7 in PIP3-induced EMT, lung cancer cells were transfected with empty vector, *pBio-PHB^WT^*, *pBio-PHB^T258I^* or *pBio-PHB^Y259F^* and then treated with PIP3. Our results showed that phospho-PHB^T258^ plays a critical role in PIP3-mediated increase of Snail. Downregulation of PHB with *pBio-PHB^T258I^* or *pBio-PHB^Y259F^*, on the other hand, did not affect Twist at all (Figure 4A).

**Figure 4:** Phospho-PHB^T258^ and MIG-7 play distinct roles in PIP3-mediated enhancement of E-cadherin suppressors in lung cancer cells (A) lung cancer cells (A549, CL1-5 and CL1-0; 2 × 10^5^/mL) were transfected with empty vector, wild-type *pBio-PHB^WT^*, mutant *pBio-PHB^T258I^* or *pBio-PHB^Y259F^* plasmid constructs for 48 hours and then treated with PIP3 (5 μM) for 24 hours. (B) cells were transfected with control scrambled siRNA (−*siIKKα/β*, −*siRaf-1*, or −*MIG7-1*), IKKα/β siRNA (*+siIKKα/β*), siRaf-1 siRNA (*+siRaf-1*), *pBio-PHB^T258I^*, or MIG-7-1 siRNA (+*siMIG7-1*) for 48 hours and then treated with PIP3 (5 μg/mL) for 24 hours as indicated. Proteins were determined by immunoblotting. Blots are representative of three independent experiments.

Since phospho-PHB^T258^ is associated with the IKKα/β (Figure 3C, 3D, Supplementary Figure 3A and 4B) and Raf-1 signaling pathways [9], we further examined whether PIP3 increases Snail and EMT via the IKKα/β and/or Raf-1 signaling pathway. Knockdown of IKKα/β with siRNA (*siIKKα/β*) abolished PIP3-induced IKKα/β and phospho-IKKα/β^S176/189^ and partially modulated the effects of PIP3 on Snail and EMT (Figure 4B, left panel). Knockdown of Raf-1 with Raf-1 siRNA (*siRaf-1*) abolished PIP3-induced Raf-1 and phospho-Raf-1^S338^ and partially modulated the effects of PIP-3 on Snail and EMT (Figure 4B, left panel). A combination of *siIKKα/β* and *siRaf-1* abolished PIP3-induced Snail and modulated PIP3-mediated EMT better than either *siIKKα/β* or *siRaf-1* alone (Figure 4B, left panel), indicating that PIP3 increases Snail via activation of phosphorylated IKKα/β complexes and Raf-1 signaling pathways.

Neither PHB nor IKK/Raf affects Twist (Figure 4A and 4B) which has previously been shown to be MIG-7 dependent [8]. Knockdown of MIG-7 with siRNA of MIG-7 (*siMIG7-*1 or *siMIG7-2*) inhibited the PIP3-induced ZEB1 and Twist, but only partially attenuated EMT (Figure 4B right panel and Supplementary Figure 5A). PIP3-mediated ZEB1, Snail, Twist and EMT were greatly diminished only after downregulating both phospho-PHB^T258^ and MIG-7 with *pBio-PHB^T258I^* and *siMIG7* (*siMIG7-1* or *siMIG7-2*) (Figure 4B, right panel and Supplementary Figure 5A).

### Downregulation of MIG-7 and phospho-PHB has an additive effect on attenuation of lung cancer migration/invasion *in vitro* and colonization/metastasis *in vivo*

Further examination of the effects of phospho-PHB^T258^ and MIG-7 showed that dominant negative *phospho-PHB* (e.g., the *pBio-PHB^T258I^* and *pBio-PHB^Y259F^* mutants) caused only partial modulation (40-50%) of PIP3-mediated MMP2 and migration/invasion *in vitro* (Figure 5A). The effect of PIP3 on MMP2 and migration/invasion of lung cancer cells was almost completely diminished after combination treatment with *pBio-PHB^T258I^* and *siMIG7* (Figure 5B and Supplementary Figure 5), indicating that phospho-PHB^T258^ and MIG-7 are each responsible for part rather than all of the effects on cancer MMP2 activity and migration/invasion.

**Figure 5:** PIP3 increases MMP2 and migration/invasion of lung cancer cells via both phospho-PHB^T258^ and MIG-7 Cells were examined by zymography for MMP activity and transwell assay for cell migration and invasion as described in Materials and Methods. (A and B) cells were transfected with control vector (EV), *pBio-PHB^WT^*, *pBio-PHB^T258I^*, *pBio-PHB^Y259F^*, control scrambled siRNA (−*MIG7-1*) or *siMIG7-1* for 48 hours and then treated with or without PIP3 (5 μM) for 24 hours as indicated. Data represent means ± SD of 3 independent experiments; *, *P* < 0.05 and **, *P* < 0.01 by t test.

To investigate the effects of downregulating both MIG-7 and phospho-PHB on seeding and colonization of lung cancer cells *in vivo*, we generated CL1-5^EV-GL^, CL1-5^shCont-GL^, CL1-5^bPHBT258I-GL^, CL1-5^shMIG7-1-GL^, CL1-5^shMIG7-2-GL^, CL1-5^bPHBT258I/shMIG7-1-GL^ and CL1-5^bPHBT258I/shMIG7-2-GL^ cells stably expressing not only green fluorescent protein and luciferase (GL) but also empty vector (EV), control shRNA (shCont), bio-PHB^T258I^ (bPHBT258I), MIG7-1 shRNA (shMIG7-1), MIG7-2 shRNA (shMIG7-2), bPHBT258I and shMIG7-1 (bPHBT258I/shMIG7-1), or bPHBT258I and shMIG7-2 (bPHBT258I/shMIG7-2), as indicated (Supplementary Figure 6A). Proliferation assay showed that all cells grew and duplicated at similar rate (Supplementary Figure 6B). Inoculation of mice with these cells, however, demonstrated that on day 49 post-inoculation CL1-5^EV-GL^- and CL1-5^shCont-GL^-bearing mice developed more tumor nodules than mice bearing PHB^T258^ or MIG-7-downregulated CL1-5 such as CL1-5^bPHBT258I-GL^, CL1-5^shMIG7-1-GL^ or CL1-5^shMIG7-2-GL^, whereas mice bearing CL1-5 with downregulation of both PHB^T258^ and MIG-7 (CL1-5^bPHBT258I/shMIG7-1-GL^, or CL1-5^bPHBT258I/shMIG7-2-GL^) did not develop any detectable tumors (Figure 6A and 6B). These results were in agreement with the migration/invasive capability of these cells *in vitro* (Supplementary Figure 6C). There was more downregulation of Ki67 and upregulation of E-cadherin in mice inoculated with CL1-5^bPHBT258I-GL^, CL1-5^shMIG7-1-GL^, CL1-5^shMIG7-2-GL^, CL1-5^bPHBT258I/shMIG7-1-GL^ and CL1-5^bPHBT258I/shMIG7-2-GL^ cells than in those inoculated with CL1-5^EV-GL^ or CL1-5^shCont-GL^ (Figure 6C). Analysis of lung tissue lysates showed that mice implanted with CL1-5^EV-GL^ or CL1-5^shCont-GL^ had the highest EMT (Figure 6D) in comparison with the others. Interestingly, the EMT of lung tissue lysates in CL1-5^bPHBT258I/shMIG7-1-GL^ and CL1-5^bPHBT258I/shMIG7-2-GL^-inoculated mice was at a low level that was similar to tumor-free control mice (Figure 6D). Moreover, all the CL1-5^EV-GL^ or CL1-5^shCont-GL^-bearing mice and about 50-60% of CL1-5^bPHBT258I-GL^-, CL1-5^shMIG7-1-GL^- and CL1-5^shMIG7-2-GL^-bearing mice perished on day 58 post-inoculation; whereas all the CL1-5^bPHBT258I/shMIG7-1-GL^- and CL1-5^bPHBT258I/shMIG7-2-GL^-inoculated mice were all alive on day 80 post-inoculation (Figure 6E).

**Figure 6:** Downregulation of both MIG-7 and phosphorylated PHB has an additive effect on inhibition of lung cancer cell colonization/metastasis *in vivo* CL1-5^EV-GL^, CL1-5^shCont-GL^, CL1-5^bPHBT258I-GL^, CL1-5^shMIG7-1-GL^, CL1-5^shMIG7-2-GL^, CL1-5^bPHBT258I/shMIG7-1-GL^ and CL1-5^bPHBT258I/shMIG7-2-GL^ cells were generated as described in Materials and Methods. The vehicle and cells were injected respectively into tail veins of 8 groups of mice (1 × 10^6^/50 μl/mouse) in the order (1) vehicle, (2) CL1-5^EV-GL^, (3) CL1-5^shCont-GL^, (4) CL1-5^bPHBT258I-GL^, (5) CL1-5^shMIG7-1-GL^, (6) CL1-5^shMIG7-2-GL^, (7) CL1-5^bPHBT258I/shMIG7-1-GL^ and (8) CL1-5^bPHBT258I/shMIG7-2-GL^ cells. Seven weeks after cell implantation, bioluminescent images of whole body and lung as well as H&E, immunohistochemical staining and cell lysates of lung were taken. (A and B) the whole bodies of mice were detected by bioluminescent imaging and the lungs of mice were dissected from the surrounding tissue for weight and tumor nodule measurement. Data represent means ± SD of at least 3 mice of each group; *, *P* < 0.05 and **, *P* < 0.01 by t test. (C) the murine lung sections were analyzed after H&E (×40 magnification) and immunohistochemistry staining (×40 magnification; insets ×200 magnification). Data represent means ± SD of at least 3 mice of each group; *, *P* < 0.05 and **, *P* < 0.01 by t test. (D) cell lysates of 3 lung tissue samples from 3 mice in each group were extracted and analyzed by immunoblotting. Blots are representative of 3 independent experiments. (E) Mice inoculated with CL1-5^EV-GL^ and CL1-5^shCont-GL^ had a shorter mean lifespan than mice inoculated with CL1-5^bPHBT258I-GL^, CL1-5^shMIG7-1-GL^ or CL1-5^shMIG7-2-GL^ cells (43 days vs 60 days; *P* < 0.001, *n* = 6 by t test). In comparison, mice inoculated with, CL1-5^bPHBT258I/shMIG7-1-GL^ or CL1-5^bPHBT258I/shMIG7-2-GL^ cells had the longest lifespan (88 days; *P* < 0.0001, *n* = 6 by t test) in all CL1-5 xenograft mice.

## DISCUSSION

Although aberrant growth factor receptors and high levels of COX-2/PGE2 are associated with tumor angiogenesis, cancer motility and invasiveness and are correlated with poor prognosis in lung cancer [10-14, 18-21], the mechanisms of action are not fully elucidated. We recently reported that COX-2/PGE2 induces Akt/GSK-3β and wnt signaling (β-catenin/T-cell factor/lymphoid enhancer factor) to increase MIG-7 that inhibits protein phosphatase 2A (PP2A) to positively feedback on Akt/GSK-3β signaling and sustain cancer cell migration/invasion [8]. In this study, we further found that growth factors and PGE2 increased PIP3 and phospho-PHB^T258^ which played critical role in the formation of a complex of Ras, phospho-Raf-1^S338^, phospho-Akt^S473^, phospho-PHB^T258^, MEKK1 and phospho-IKKα/β^S176/180^ in the membrane rafts and elevation of phospho-NF-kB p65^S536^ leading to enhancement of COX-2 and generation of cellular PGE2 in an autocrine-like manner (Figure 2-3 and Supplementary Figure 1-4). It is possible that this type of autocrine signaling and enrichment of cellular PGE2 may have a cumulative effect producing sufficient concentration of PGE2 for lung cancer cells to survive and proliferate in metastatic sites, although this hypothesis remains to be verified.

We have recently showed that MIG-7 level was elevated at 12 hours and stayed at plateau for a long time after PGE2 treatment via Akt/GSK-3 and wnt signaling to inactivate PP2A and sustain phosphorylation of Akt and ERK [8]. In this study, we found that the upregulation of MIG-7 and the effects of MIG-7 on ZEB-1, Twist and EMT did not require the presence of active phospho-PHB^T258^ (Figure 4B, right panel). We, therefore, assert that phospho-PHB^T258^ may play a critical role in the initiation, whereas MIG-7 may play a role in long-term sustainment and augmentation of the effects of growth factors, PGE2 and PIP3 on migration/invasion of lung cancer cells (as illustrated in Figure 7).

**Figure 7:** Schematic diagram illustrates the roles of PHB and MIG-7 in regulating the effects of growth factors and PGE2 on lung cancer migration/invasion

Transcriptional suppressors of E-cadherin, notably ZEB-1, Snail and Twist regulate EMT and play a critical role in cancer invasion/metastasis [26, 27]. The mechanism of regulatory action of each E-cadherin suppressors, however, is not well delineated. In this study, we found that the increase of Snail via phospho-PHB^T258^ depended on not only the IKK/β complex but also Raf-1 signaling (Figure 4A and 4B, left panels), whereas MIG-7 was mainly associated with increase in ZEB-1 and Twist (Figure 4B, right panel). In addition, growth factors and PGE2 induced PIP3 and phospho-PHB^T258^ as well as MIG-7 with distinct temporal patterns [8] (Figure 1 and 2). Combined attenuation of phospho-PHB^T258^ and MIG-7 blocked EMT (Figure 4B, right panel) leading to abolishment of lung cancer cells migration/invasion (Figure 5B and Supplementary Figure 5). These results demonstrated that there are several E-cadherin suppressors each of which is regulated by more than one pathway. Whether each of these transcriptional suppressors is responsible for regulating EMT and cell migration/invasion at different cellular stages and whether each act coordinately with others under physiological or pathological conditions remains to be elucidated.

Growth factors and PGE2-mediated elevation of PIP3 is associated with the induction of Akt/IKKα/β/IκB/NF-kB signaling and COX-2 [22, 23], but the underlying molecular mechanism is not fully elucidated. We found that PIP3 increased phospho-IKKα/β^S176/180^ together with MEKK1 but not NIK in the raft domain (Figure 3B and 3C). Such effect of PIP3 was dependent on the presence of active Akt and PHB (Figure 3 and Supplementary Figure 3A). PIP3 also increased phospho-NF-kB p65^S536^ and COX-2/PGE2 and this increase was attenuated by downregulating phospho-PHB with phospho-PHB^T258I/Y259F^ (Supplementary Figure 4A). These results indicate that PIP3 activates Akt and PHB that in turns activates MEKK1 in the raft domain to induce IKKα/β/IκB/NF-kB signaling as well as phospho-NF-kB p65^S536^ and COX-2/PGE2.

Treatment of cells with or without *siIKKα/β* and *siRaf-1* demonstrated that phospho-NF-kB p65^S536^ and COX-2 were selectively attenuated by IKKα/β knockdown whereas Raf-1 knockdown diminished phosphorylation of ERK^T185/Y187^, MYPT1^T696^ and MLC2^T18/S19^ but not COX-2 (Supplementary Figure 7B). It is likely that enhancement of COX-2 is MEKK1 and IKKα/β^S176/180^ dependent. Raf-1, on the other hand, regulated cell migration mainly via MYPT1/MLC2 pathway as we have previously shown [9] rather than via enhancement of COX-2 expression (as illustrated in Figure 7).

Over-activation of EGFR, PI3K/Akt, and RAS or loss of p53 protection is frequently found and associated with poor prognosis in a variety of human lung cancers [28]. Among the lung cancer cell lines that we have examined so far, A549 has oncogenic KRAS [29], whereas H1299 is null in p53 [30]. Both cell lines were affected by downregulation of phospho-PHB^T258^ and MIG-7 [8] (Figure 4, 5 and Supplementary Figure 5). In addition, we found that EGF, HGF and IGF-1 all increased PIP3 and phospho-Akt whose effects on lung cancer migration/invasion were attenuated by downregulating phospho-PHB^T258^ and MIG-7 too (Figure 4, 5 and Supplementary Figure 5). Our results thus suggested that phospho-PHB^T258^ and MIG-7 likely play critical role in invasion/metastasis of not just a single minor subtype but the majority, if not all kinds, of lung cancers.

Combination targeted therapy, if designed properly to target several complementary key effectors, can result in fewer adversary responses and less drug resistance, leading to more effectiveness than traditional targeted therapy that interferes with only a specific molecule and/or pathway. In this study, we showed that levels of MIG-7 protein and plasma membrane-associated PHB correlated with advanced stages of cancers in human lung tumor tissues (Figure 1). Downregulation of phospho-PHB^T258^ and MIG-7 was significantly more effective than downregulation of either phospho-PHB^T258^ or MIG-7 alone in decreasing cancer invasion/metastasis and increasing the disease-free as well as overall survival of human lung cancer xenograft mice (Figure 6). It will be of interest to examine whether combination targeting of phospho-PHB^T258^ and MIG-7 will be beneficial for treating metastatic lung cancer patients.

## MATERIALS AND METHODS

### Cell culture

Cells were maintained in DMEM or RPMI medium (GibcoBRL Life Technologies, Grand Island, NY) supplemented with 10% fetal bovine serum (FBS; GibcoBRL Life Technologies) and 1% penicillin-streptomycin-neomycin (GibcoBRL Life Technologies). Unless specified otherwise, 2 × 10^5^/mL cells were used in each experiment. The lung cancer A549 (ATCC: CCL-185) cell line was certified by the Food Industry Research and Development Institute (Hsinchu, Taiwan). CL1-0 and CL1-5 were obtained as described previously [31]. *In vitro* cell proliferation was measured by WST-1 assay according to the manufacturer's instructions (Roche, Mannheim, Germany).

### Generation of *pD-PHB*, *pBio-PHB* and PHB mutants

Human PHB was cloned in pcDNA6/BioEase-DEST vector (Invitrogen) to generate the plasmid *pBio-PHB* which expressed PHB tagged with biotin. The PHB mutants were produced using the QuikChange Site-directed Mutagenesis Kit (Stratagene, La Jolla, CA). *pD-PHB* was produced as described previously [9].

### Transfection of cDNA, siRNAs and shRNAs

cDNA, siRNAs and shRNAs were transfected into cell lines by GenMute siRNA Transfection Reagent (SignaGen Laboratories, Gaithersburg, MD) according to the manufacturer's protocol. The expression of target proteins in the transfected cells was determined 48 hours after transfection, unless specified otherwise. The cDNA- and shRNA-transduced cells were selected by G418 (Sigma-Aldrich, St. Louis, MO).

### Measurement of PGE2

The level of cellular and secreted PGE2 was measured using a commercially available PGE2 EIA assay kit (Amersham, Arlington Heights, IL).

### Determination of PIP3

Phospholipids were extracted and PIP3 levels were measured by ELISA using PIP3 Mass ELISA Kit (Echelon Biotechnology).

### Extraction of membrane raft proteins

Membrane raft proteins were extracted as described previously [9].

### Immunoblotting, immunoprecipitation and gelatin zymographic analysis

Gelatinolytic activities of MMP-2 and MMP-9, immunoprecipitation and immunoblotting were performed as described previously [8, 9].

### Migration and invasion assays

Migration and invasion assays were performed *in vitro* as described previously [8, 9].

### Ras activity assay

Ras activity was measured using the Ras Activation Assay Kit (Upstate Biotechnology) according to the manufacturer's instructions.

### Preparation of pCMV-GFP/luciferase-lentivirus and establishment of stable cell lines

CL1-5^GL^ cells were produced by infecting CL1-5 cells with cytomegalovirus promoter (pCMV)-GFP/luciferase-lentivirus as described previously [8]. CL1-5^GL^ cell lines were transfected with control shRNA, MIG7-1 shRNA, MIG7-2 shRNA, pBio-vector plasmid and *pBio-PHB^T258I^* plasmid separately and selected with G418 (400 μg/mL) to produce CL1-5^shCont-GL^, CL1-5^shMIG7-1-GL^, CL1-5^shMIG7-2-GL^, CL1-5^EV-GL^ and CL1-5^bPHBT258I-GL^ stable cell lines. CL1-5^shMIG7-1-GL^ and CL1-5^shMIG7-2-GL^ cells were then transfected with *pBio-PHB^T258I^* plasmid to produce CL1-5^bPHBT258I/shMIG7-1-GL^ and CL1-5^bPHBT258I/shMIG7-2-GL^ cells. The expression levels and effects of MIG-7 shRNA and *pBio-PHB^T258I^* in each stable cell line were analyzed by immunoblot analysis, proliferation assay, migration and invasion assay *in vitro*.

### Experimental xenograft murine metastasis model

Male severe combined immunodeficiency (SCID) mice (C.B17/lcr-Prkdc ^scid^/CrlNarl) were purchased from the National Laboratory Animal Center (Taipei, Taiwan). All animal care and *in vivo* experiments were performed in compliance with the guidelines of the Academia Sinica Institutional Animal Care and Utilization Committee. Mice (*n* = 9/group) were implanted with 50 μL RPMI medium as control (vehicle) or 1 × 10^6^/50 μL lung tumor cells on day 0 by lateral tail vein injection. Metastatic progression was monitored weekly and quantified using a noninvasive bioluminescence IVIS Imaging System (Xenogen, Alameda, CA) as described previously [8]. Forty-nine days after injection, three mice were killed for necropsy and the other 6 mice were kept for survival studies. The percentage of animal survival in each group was routinely recorded.

### Immunohistochemistry and histopathology examination

Immunohistochemistry and histopathology analyses as well as immunohistochemical scoring were performed as described previously [8, 9]. MIG-7 scores were generated by the percentage positive cells multiplied by stain intensity (Score 0 = negative, 1-2 = weak, 3-4 = moderate, 5-6 = strong). The images were scanned into a digital format by Scanscope XT system (Aperio Technologies, Vista, CA) and analyzed using Aperio ImageScope 9.1 software (Aperio Technologies).

### Statistics

All statistical comparisons were made with two-tailed tests. The survival time was assessed using Kaplan-Meier curves and tested for significance by the log-rank test. Statistical evaluation was performed using GraphPad Prism version 5.0 for Microsoft Windows (GraphPad Software, La Jolla, CA). Differences between groups were considered statistically significant at P values of less than 0.05 or 0.01.

## SUPPLEMENTARY MATERIAL AND FIGURES



## References

[1] Fidler IJ (2003). The pathogenesis of cancer metastasis: the ‘seed and soil’ hypothesis revisited. Nature reviews Cancer.

[2] Liotta LA, Stetler-Stevenson WG (1991). Tumor invasion and metastasis: an imbalance of positive and negative regulation. Cancer research.

[3] Sun S, Schiller JH, Spinola M, Minna JD (2007). New molecularly targeted therapies for lung cancer. The Journal of clinical investigation.

[4] Perlikos F, Harrington KJ, Syrigos KN (2013). Key molecular mechanisms in lung cancer invasion and metastasis: a comprehensive review. Critical reviews in oncology/hematology.

[5] Crouch S, Spidel CS, Lindsey JS (2004). HGF and ligation of alphavbeta5 integrin induce a novel, cancer cell-specific gene expression required for cell scattering. Experimental cell research.

[6] Petty AP, Garman KL, Winn VD, Spidel CM, Lindsey JS (2007). Overexpression of carcinoma and embryonic cytotrophoblast cell-specific Mig-7 induces invasion and vessel-like structure formation. The American journal of pathology.

[7] Phillips TM, Lindsey JS (2005). Carcinoma cell-specific Mig-7: a new potential marker for circulating and migrating cancer cells. Oncology reports.

[8] Ho MY, Liang SM, Hung SW, Liang CM (2013). MIG-7 controls COX-2/PGE2-mediated lung cancer metastasis. Cancer research.

[9] Chiu CF, Ho MY, Peng JM, Hung SW, Lee WH, Liang CM, Liang SM (2013). Raf activation by Ras and promotion of cellular metastasis require phosphorylation of prohibitin in the raft domain of the plasma membrane. Oncogene.

[10] Brown JR, DuBois RN (2004). Cyclooxygenase as a target in lung cancer. Clinical cancer research : an official journal of the American Association for Cancer Research.

[11] Castelao JE, Bart RD, DiPerna CA, Sievers EM, Bremner RM (2003). Lung cancer and cyclooxygenase-2. The Annals of thoracic surgery.

[12] Hida T, Yatabe Y, Achiwa H, Muramatsu H, Kozaki K, Nakamura S, Ogawa M, Mitsudomi T, Sugiura T, Takahashi T (1998). Increased expression of cyclooxygenase 2 occurs frequently in human lung cancers, specifically in adenocarcinomas. Cancer research.

[13] Wolff H, Saukkonen K, Anttila S, Karjalainen A, Vainio H, Ristimaki A (1998). Expression of cyclooxygenase-2 in human lung carcinoma. Cancer research.

[14] Chell S, Kaidi A, Williams AC, Paraskeva C (2006). Mediators of PGE2 synthesis and signalling downstream of COX-2 represent potential targets for the prevention/treatment of colorectal cancer. Biochimica et biophysica acta.

[15] Church RJ, Jania LA, Koller BH (2012). Prostaglandin E(2) produced by the lung augments the effector phase of allergic inflammation. J Immunol.

[16] Davis R, Rizwani W, Banerjee S, Kovacs M, Haura E, Coppola D, Chellappan S (2009). Nicotine promotes tumor growth and metastasis in mouse models of lung cancer. PloS one.

[17] Moraitis D, Du B, De Lorenzo MS, Boyle JO, Weksler BB, Cohen EG, Carew JF, Altorki NK, Kopelovich L, Subbaramaiah K, Dannenberg AJ (2005). Levels of cyclooxygenase-2 are increased in the oral mucosa of smokers: evidence for the role of epidermal growth factor receptor and its ligands. Cancer research.

[18] Wang D, Dubois RN (2010). Eicosanoids and cancer. Nature reviews Cancer.

[19] Bredin CG, Liu Z, Klominek J (2003). Growth factor-enhanced expression and activity of matrix metalloproteases in human non-small cell lung cancer cell lines. Anticancer research.

[20] Amann J, Kalyankrishna S, Massion PP, Ohm JE, Girard L, Shigematsu H, Peyton M, Juroske D, Huang Y, Stuart Salmon J, Kim YH, Pollack JR, Yanagisawa K, Gazdar A, Minna JD, Kurie JM (2005). Aberrant epidermal growth factor receptor signaling and enhanced sensitivity to EGFR inhibitors in lung cancer. Cancer research.

[21] Yin M, Guan X, Liao Z, Wei Q (2009). Insulin-like growth factor-1 receptor-targeted therapy for non-small cell lung cancer: a mini review. American journal of translational research.

[22] Hannigan G, Troussard AA, Dedhar S (2005). Integrin-linked kinase: a cancer therapeutic target unique among its ILK. Nature reviews Cancer.

[23] Hsu HC, Fong YC, Chang CS, Hsu CJ, Hsu SF, Lin JG, Fu WM, Yang RS, Tang CH (2007). Ultrasound induces cyclooxygenase-2 expression through integrin, integrin-linked kinase, Akt, NF-kappaB and p300 pathway in human chondrocytes. Cellular signalling.

[24] Shishodia S, Koul D, Aggarwal BB (2004). Cyclooxygenase (COX)-2 inhibitor celecoxib abrogates TNF-induced NF-kappa B activation through inhibition of activation of I kappa B alpha kinase and Akt in human non-small cell lung carcinoma: correlation with suppression of COX-2 synthesis. J Immunol.

[25] Nakano H, Shindo M, Sakon S, Nishinaka S, Mihara M, Yagita H, Okumura K (1998). Differential regulation of IkappaB kinase alpha and beta by two upstream kinases, NF-kappaB-inducing kinase and mitogen-activated protein kinase/ERK kinase kinase-1. Proceedings of the National Academy of Sciences of the United States of America.

[26] Yang J, Weinberg RA (2008). Epithelial-mesenchymal transition: at the crossroads of development and tumor metastasis. Developmental cell.

[27] Zheng H, Kang Y (2013). Multilayer control of the EMT master regulators. Oncogene.

[28] Cooper WA, Lam DC, O'Toole SA, Minna JD (2013). Molecular biology of lung cancer. Journal of thoracic disease.

[29] Choi EJ, Ryu YK, Kim SY, Wu HG, Kim JS, Kim IH, Kim IA (2010). Targeting epidermal growth factor receptor-associated signaling pathways in non-small cell lung cancer cells: implication in radiation response. Molecular cancer research : MCR.

[30] Scian MJ, Stagliano KE, Ellis MA, Hassan S, Bowman M, Miles MF, Deb SP, Deb S (2004). Modulation of gene expression by tumor-derived p53 mutants. Cancer research.

[31] Chu YW, Yang PC, Yang SC, Shyu YC, Hendrix MJ, Wu R, Wu CW (1997). Selection of invasive and metastatic subpopulations from a human lung adenocarcinoma cell line. American journal of respiratory cell and molecular biology.

[32] Delcommenne M, Tan C, Gray V, Rue L, Woodgett J, Dedhar S (1998). Phosphoinositide-3-OH kinase-dependent regulation of glycogen synthase kinase 3 and protein kinase B/AKT by the integrin-linked kinase. Proceedings of the National Academy of Sciences of the United States of America.

